The article "Expression of CX3CL1 and CCL28 in Spinal Metastases of Lung Adenocarcinoma and Their Correlation with Clinical Features and Prognosis" was retracted in 2023. Reasons: suspected computer-generated content; unreliable results or conclusions; concerns about the data; concerns about the results or conclusions.

# Expression of CX3CL1 and CCL28 in Spinal Metastases of Lung Adenocarcinoma and Their Correlation with Clinical Features and Prognosis

**DOI:** 10.1155/2022/2580419

**Published:** 2022-04-21

**Authors:** Shuguang Li, Shuai Liu, Jianjun Xun, Feifei Zhao

**Affiliations:** ^1^Department of Radiation Oncology, the Fourth Hospital of Hebei Medical University, Shijiazhuang 050011, Hebei, China; ^2^Department of Orthopedics, the Fourth Hospital of Hebei Medical University, Shijiazhuang 050011, Hebei, China

## Abstract

Lung adenocarcinoma is the most common non-small-cell lung cancer. In this paper, we aim to investigate the expression of chemokine ligand 1 (cx3cl1) and chemokine ligand 28 (CCL28) in spinal metastases of lung adenocarcinoma and their correlation with clinical features and prognosis. We analyzed the clinical data of 40 patients with lung adenocarcinoma and spinal metastases who underwent surgery in our hospital from January 2018 to January 2021 retrospectively. The expression levels of cx3cl1 and CCL28 in bone metastases were detected by immunohistochemistry, and the staining results were sorted and classified. Combined with the follow-up results and clinicopathological data, we statistically analyzed the expression of cx3cl1 and CCL28 in spinal bone metastases and their correlation with prognosis. Among the 40 patients with spinal metastasis of lung adenocarcinoma, 7 cases were strongly positive for cx3cl1, 25 cases were moderately positive, and 8 cases were weakly positive and negative. CCL28 was strongly positive in 9 cases, moderately positive in 26 cases, weakly positive and negative in 5 cases. The expression of cx3cl1 was correlated with ECOG score (*P* = 0.005) and visceral organ metastasis (*P* = 0.004), but not with age, sex, and the number of bone metastases (*P* > 0.05). The expression of CCL28 was correlated with ECOG score (*P* = 0.022) and visceral organ metastasis (*P* = 0.003), but not with age, sex, and the number of bone metastases (*P* > 0.05). The OS of patients with strong cx3cl1 positive was significantly shorter than that of patients with medium positive and weak positive (*P* < 0.001). The survival time was 10, 7, and 4 months, respectively. The OS of patients with strong positive CCL28 was significantly shorter than that of patients with medium positive and weak positive CCL28 (*P* = 0.004). The survival time was 12, 8, and 4 months, respectively. Univariate analysis showed that ECOG score (*P* < 0.001), chemotherapy (*P* = 0.032), visceral organ metastasis (*P* = 0.002), cx3cl1 expression (*P* < 0.001), and CCL28 expression (*P* = 0.004) were the risk factors of OS. Cox regression analysis showed that the expression of cx3cl1 was an independent risk factor for OS in patients with spinal metastasis of lung adenocarcinoma (*P* = 0.044). Cx3cl1 and CCL28 were highly/strongly positive in spinal metastases of lung adenocarcinoma. The level of cx3cl1 can be used as an index to judge the clinical prognosis of patients with spinal metastasis of lung adenocarcinoma, which can better reflect the prognosis of patients than CCL28.

The article "Expression of CX3CL1 and CCL28 in Spinal Metastases of Lung Adenocarcinoma and Their Correlation with Clinical Features and Prognosis" was retracted in 2023. Reasons: suspected computer-generated content; unreliable results or conclusions; concerns about the data; concerns about the results or conclusions.

## 1. Introduction

Spinal bone metastasis of lung adenocarcinoma refers to the disease that primary lung adenocarcinoma metastasizes to the spine through blood or lymph. For spinal bone metastasis, the self-regulation and remodeling of the lesion microenvironment are particularly important for all kinds of tumor metastasis. Therefore, it can be speculated that some cytokines or inflammatory mediators in the microenvironment of spinal metastasis of lung adenocarcinoma may be involved in the process of metastasis [1].

Studies have found that cx3cll and its receptor are expressed in many different types of malignant tumors and play an important role in tumor proliferation, invasion, and migration [2]. In the mammary cancer mouse model, the induction of CX3CL1 seems to increase the infiltration of CX3CR1+ macrophages and tumor angiogenesis. CX3CR1 is also overexpressed in the spinal metastasis of breast cancer, while CX3CL1 is expressed in the cancellous bone. This indicates that malignant cells expressing CX3CR1 may be attracted to the gradient direction of CX3CL1 to bone [3]. CCL28 is a chemokine constitutively expressed in a variety of mucosal tissues and an important mediator of mucosal immunity [4]. Studies have found that CCL28 is the only hypoxia-inducible chemokine in lung adenocarcinoma cells. CCL28 can promote the tubular formation, migration, and proliferation of endothelial cells. The lung adenocarcinoma cells with high expression of CCL28 grow faster and have a higher vascular density, while the lung adenocarcinoma cells with downregulated expression of CCL28 have lower tumor formation rate and lower vascular density [5]. CCL28 is not only highly expressed in a variety of tumor tissues, such as liver cancer, prostate cancer, and ovarian cancer, but can also participate in the regulation of inflammation and immunity by binding to the corresponding receptors. Studies have shown that the chemokine axis cx3cl1-cx3cr1 can promote the migration and invasion of various tumors. Cx3cl1-cx3cr1 can promote osteosarcoma metastasis by activating PI3K/Akt/NF KB. Other studies have found that cx3cl1-cx3cr1 can regulate the invasion, proliferation, and migration of prostate cancer through the PI3K/Akt pathway [6]. In addition, CX3CL1-CX3CR1 can also regulate the development of breast cancer by activating the MAPK/ERK signaling pathway [7]. These effects may further promote the proliferation, invasion, and migration of tumor cells, inhibit tumor cell apoptosis, and stimulate tumor-related angiogenesis to promote the infiltration, diffusion, and further metastasis of tumor cells.

The article "Expression of CX3CL1 and CCL28 in Spinal Metastases of Lung Adenocarcinoma and Their Correlation with Clinical Features and Prognosis" was retracted in 2023. Reasons: suspected computer-generated content; unreliable results or conclusions; concerns about the data; concerns about the results or conclusions.

By analyzing the expression of spinal bone metastasis in lung adenocarcinoma, this paper further explores the relationship between clinical and pathological features, influencing factors, and prognosis. And we detected the expression levels of cx3cl1 and CCL28 in bone metastases by immunohistochemistry.

## 2. Materials and Methods

### 2.1. Research Object

40 cases of lung adenocarcinoma and spinal metastasis confirmed by postoperative pathology in the fourth hospital of Hebei Medical University from January 2018 to January 2020 were collected. The inclusion criteria were as follows: after surgical treatment and independent review by pathologists in our hospital, the diagnosis was confirmed by immunohistochemical staining. Patients aged between 43 and 79. Preoperative radiotherapy and chemotherapy were not performed. The patient's case data and follow-up data are complete. The experiment was with the informed consent of all patients. And we were reviewed by the hospital ethics committee. The exclusion criteria were as follows: (1) patients with incomplete case data. (2) Death from noncancerous causes. (3) No second primary tumor, serious other system dysfunction. And we collected the patients' gender, age, number of bone metastases, chemotherapy or not, ECOG score, visceral metastasis or not, and the expression levels of cx3cl1 and CCL28 in metastatic lesions. In addition, we followed up all patients by outpatient follow-up or telephone. The follow-up time was 3 ∼ 14 months, and the deadline was January 2021. The endpoint was death from lung adenocarcinoma or its complications. Overall survival refers to the time from surgery to patient death.

### 2.2. Immunohistochemical Staining

Rabbit polyclonal antibody cx3cl1: model (ab25088) and rabbit polyclonal antibody CCL28: model (ab232837) were purchased from Abcam, Cambridge, UK. All the specimens were fixed in formalin and made into paraffin sections by the routine process. All the sections were fully baked for immunohistochemical staining. PBS instead of the primary antibody was used as the negative control, known positive sections were used as the positive control, and the ratio of cell staining intensity to the number of positive cells was used for the comprehensive score.

The cytoplasm from light yellow to dark brown was used as the marker of positive cells, which was 5 times higher (× 200) count the positive cells in the visual field, and calculate the positive rate: 0–5% is 0, 6%–25% is 1, 26%–50% is 2, 51%–75% is 3, 76%–100% is 4. According to the staining conditions of most cells, the staining intensity standard is set, including 3 points for tan, 2 points for brown, 1 point for light yellow, and 0 points for nonstaining. Finally, the product of positive cell percentage and staining intensity score was calculated, and the total score was (-): 0; (+): 1–4 points; (++): 5–8 points; (++ +): 9–12 points. Score ≥5 was defined as medium/high positive expression of cx3cl1 or CCL28 in tumor cells.

The article "Expression of CX3CL1 and CCL28 in Spinal Metastases of Lung Adenocarcinoma and Their Correlation with Clinical Features and Prognosis" was retracted in 2023. Reasons: suspected computer-generated content; unreliable results or conclusions; concerns about the data; concerns about the results or conclusions.

### 2.3. Statistical Analysis

SPSS 26.0 software was used for statistical analysis. If the measurement data meet the normal distribution and homogeneity of variance, a *t*-test shall be used. Otherwise, a nonparametric test shall be used. Categorical variables are used *χ* 2 test or Fisher test; the Kaplan–Meier method was used for the survival curve, and the logrank test was used for intergroup comparison. The Cox risk ratio model was used in univariate and multivariate survival analysis; the difference was statistically significant (*P* < 0.05).

At the same time [8–11]: the number of bone metastases and ECOG score are prognostic factors for bone metastases of lung cancer. The survival time of patients with single bone metastasis is longer than that of patients with multiple bone metastases. Multiple bone metastases usually indicate high activity and malignancy of tumor cells with poor prognosis. Clinical tips: timely and effective treatment after diagnosis of bone metastasis is the key to prolong survival, which is consistent with whether chemotherapy affects the prognosis of patients.

## 3. Results

### 3.1. Expression of cx3cl1 and CCL28 in Spinal Metastasis of Lung Adenocarcinoma

Among 40 patients with bone metastasis of lung adenocarcinoma, 7 cases were strongly positive for cx3cl1, 25 cases were moderately positive, and 8 cases were weakly positive and negative. The moderate/strong positive rate of cx3cl1 in patients with bone metastasis of lung adenocarcinoma was 80%. CCL28 was strongly positive in 9 cases, moderately positive in 26 cases, weakly positive and negative in 5 cases. The medium/high positive rate of CCL28 was 87.5%.  Figure 1(a)–1(c) show the low, medium, and high expression of cx3cl1 in spinal metastasis of lung adenocarcinoma respectively.  Figure 1(d)–1(f) show the low, medium and high expression of CCL28, respectively, in spinal metastasis of lung adenocarcinoma.

Note: scale bar: 50/25um, X200.

### 3.2. Correlation between Different Expression Levels of cx3cl1 and CCL28 and Other Clinical Data

As shown in Table 1, the expression levels of cx3cl1 and CCL28 in 40 patients with spinal bone metastasis of lung adenocarcinoma were significantly correlated with ECOG score (*P* = 0.005) and visceral organ metastasis (*P* = 0.004), but not with age, gender, number of bone metastasis, and chemotherapy (*P* > 0.05).

The article "Expression of CX3CL1 and CCL28 in Spinal Metastases of Lung Adenocarcinoma and Their Correlation with Clinical Features and Prognosis" was retracted in 2023. Reasons: suspected computer-generated content; unreliable results or conclusions; concerns about the data; concerns about the results or conclusions.

### 3.3. Correlation between the Expression of cx3cl1 and CCL28 in Spinal Metastasis of Lung Adenocarcinoma and Prognosis

Univariate analysis: age, gender, and the number of bone metastases had no correlation with OS in patients with bone metastases of lung adenocarcinoma (*P* > 0.05), while ECOG score [*x*2 = 12.790, *P* < 0.001], chemotherapy or not [*x*2 = 4.622, *P* < 0.05], and visceral organ metastasis [*x*2 = 10.007, *P* < 0.05] were risk factors affecting OS (Table 2). The relationship with OS was shown by the Kaplan–Meier method.  Figure 2(a)–2(e) shows the plot of cx3cl1 expression, CCL28 expression, ECOG score, internal organs, and postoperative chemotherapy, respectively.

Cox multivariate regression analysis showed that age, gender, number of bone metastases, ECOG score, chemotherapy or not, metastasis of internal organs, and CCL28 expression had no significant relationship with the overall survival time. The expression of cx3cl1 [*P* = 0.044, HR = 0.283 (0.08 ∼ 0.9)] was significantly correlated with the overall survival time of patients (Table 3).

## 4. Discussion

Among various pathological types, adenocarcinoma is also the most common type of bone metastasis, and the most common site of bone metastasis is the spine. Migration and invasion can occur in various organs in the advanced stage of cancer, which is the main cause of treatment failure and patient death, which indicates a poor prognosis. Therefore, it is very important to determine the prognostic factors. At present, there are few studies on the spinal metastasis of human lung adenocarcinoma at home and abroad.

In this study, the expression levels of cx3cl1 and CCL28 in the metastatic lesions of patients with spinal metastasis of lung adenocarcinoma were detected by immunohistochemical method. It was found that in 40 patients included in the study, the medium/high expression rate of cx3cl1 was 80%, and the medium/high expression rate of CCL28 was 87.5%. The expression of cx3cl1 and CCL28 was related to ECOG score (*P* = 0.005) and visceral organ metastasis. Univariate analysis showed that age, gender, and the number of bone metastases had no correlation with the overall survival time of patients with spinal bone metastasis of lung adenocarcinoma (*P* > 0.05), while ECOG score [*X*^2^ = 7.681, *P* < 0.05], chemotherapy or not [*X*^2^ = 4.622, *P* < 0.05], and visceral organ metastasis [*X*^2^ = 10.007, *P* < 0.05] all had significant effects on the survival time of patients. The Cox multivariate regression analysis showed that age, gender, number of bone metastases, ECOG score, chemotherapy or not, whether internal organs metastasized or not, and CCL28 expression had no statistical significance on the overall survival of patients. Only the expression of cx3cl1 [*P* = 0.044, HR = 0.283 (0.083 ∼ 0.965)] had a significant impact on the overall survival of patients. Although the results do not show that CCL28 is an independent prognostic factor for spinal metastasis of lung adenocarcinoma, cx3cl1 can significantly affect the prognosis of patients with spinal metastasis of lung adenocarcinoma. It is reported that [8] the survival time of patients with single bone metastasis is better than that of patients with multiple bone metastases, and some studies have found that there is no significant difference in survival expectation between patients with single bone metastasis and patients with multiple bone metastases.

The article "Expression of CX3CL1 and CCL28 in Spinal Metastases of Lung Adenocarcinoma and Their Correlation with Clinical Features and Prognosis" was retracted in 2023. Reasons: suspected computer-generated content; unreliable results or conclusions; concerns about the data; concerns about the results or conclusions.

However, the number of bone metastases is not a significant prognostic factor when multivariate analysis of chemoradiotherapy response status is carried out at the same time. This suggests that patients with multiple bone metastases can benefit from radiotherapy and chemotherapy. The higher the ECOG score, the worse the overall health of cancer patients. They have poor tolerance to radiotherapy and chemotherapy, so they do not benefit much from treatment. Patients have an increased risk of prognosis. The ECOG performance score is the quantification of the overall health status and activities of daily living of cancer patients. A higher ECOG score indicates that cancer patients have a poor overall health. They usually have poor tolerance to radiotherapy and chemotherapy and benefit little from treatment. In univariate analysis, the survival time of patients with low scores was much longer than that of patients with high scores. Therefore, the ECOG score is another prognostic factor for bone metastasis of lung cancer. This is also consistent with our conclusion. Although we used univariate analysis to suggest that ECOG, chemotherapy, and visceral metastasis all have an impact on the survival of patients, multivariate analysis showed that only the expression of cx3cl1 had statistical significance on survival, which we need to further analyze. At the same time, univariate regression analysis showed that the expression of cx3cl1 (*P* < 0.001) and CCL28 (*P* = 0.004) in spinal metastases was significantly correlated with OS, and with the increase of the expression of cx3cl1 and CCL28, the overall survival of patients became shorter. In addition, the expression of cx3cl1 was positively correlated with the expression of CCL28, and the correlation coefficient was rs = 0.371, which was statistically significant (*P* < 0.05), indicating that the two factors may interact in the process of spinal bone metastasis of lung adenocarcinoma, but the specific mechanism is not clear.

The article "Expression of CX3CL1 and CCL28 in Spinal Metastases of Lung Adenocarcinoma and Their Correlation with Clinical Features and Prognosis" was retracted in 2023. Reasons: suspected computer-generated content; unreliable results or conclusions; concerns about the data; concerns about the results or conclusions.

## 5. Conclusion

In summary, the roles of CX3CL1 and CCL28 in various tumors have been extensively studied. We have found that cx3cl1 is an independent risk factor for prognosis in patients with spinal metastasis of lung adenocarcinoma. Moreover, cx3cl1 and CCL28 play a key role in the spinal metastasis of lung adenocarcinoma because of the correlation between cx3cl1 and CCL28. Our finding could bring good news to the treatment of patients.

However, it is not clear whether these factors can be used as potential diagnostic and therapeutic targets. Therefore, more experiments are still needed in the future to elaborate the effects of cx3cl1 and CCL28 on the spinal metastasis of lung adenocarcinoma [12–18].

## Figures and Tables

**Figure 1:** The expression of cx3cl1 and CCL28 in spinal metastasis of lung adenocarcinoma.

**Figure 2:** Kaplan–Meier survival analysis plotted the survival curve of variables significantly related to the prognosis of patients.

**Table 1:** Correlation between different expression levels of cx3cl1 and CCL28 and clinical data.

Characteristics			CX3CL1			*P*	CCL28			*P*
			-/+ (%)	++ (%)	+++ (%)		-/+(%)	++(%)	+++(%)	
Gender	Female	21	4 (19.0)	14 (66.7)	3 (14.3)	0.592	3 (14.3)	15 (71.4)	3 (14.3)	0.549
	Male	19	4 (21.1)	11 (57.9)	4 (21.1)		2 (10.5)	12 (63.2)	5 (26.3)	
Age (years)	≥60	30	6 (20.0)	19 (63.3)	5 (16.7)	0.688	4 (13.3)	21 (70.0)	5 (16.7)	0.633
	<60	10	2 (20.0)	6 (60.0)	2 (20.0)		1 (10.0)	6 (60.0)	3 (30.0)	
Number of bonemetastases	Single	8	3 (37.5)	3 (37.5)	2 (25.0)	0.320	4 (50.0)	2 (25.0)	2 (25.0)	0.507
	Multiple	32	5 (15.6)	22 (68.75)	5 (15.6)		1 (3.1)	25 (78.1)	6 (18.8)	
ECOG scores^*∗*^	0–2	12	6 (50.0)	4 (33.3)	2 (16.6)	0.005	4 (33.3)	6 (50.0)	2 (16.7)	0.022
	3–4	28	2 (7.1)	21 (75)	5 (17.9)		1 (3.6)	21 (75.0)	6 (21.4)	
Chemotherapy	No	17	2 (11.8)	10 (58.9)	5 (29.4)	0.428	2 (11.8)	13 (76.5)	2 (11.8)	0.646
	Yes	23	6 (26.1)	15 (65.2)	2 (8.7)		3 (13.0)	14 (60.9)	6 (26.1)	
Visceral metastasis^*∗*^	No	8	5 (62.5)	2 (25.0)	1 (12.5)	0.004	4 (50.0)	2 (25.0)	2 (25.0)	0.003
	Yes	32	3 (9.4)	23 (71.9)	6 (18.8)		1 (3.1)	25 (78.1)	6 (18.8)	

^*∗*^ *P*＜0.05, indicating statistical significance.

**Table 2:** Prognostic relevance of clinicopathological variables for overall survival.

Variables	Patients (n)	Patients (%)	Mean survival months	95% CL	*P* values
Gender					
Female	21	52.5	8.0	4.89–11.11	0.350
Male	19	47.5	7.0	5.82–8.18	

Age (years)					
<60	10	25.0	8.0	5.61–10.39	0.580
≥60	30	75.0	7.0	5.29–8.71	

Number of bone metastases					
Single	8	20.0	8.0	5.32–10.68	0.748
Multiple	32	80.0	7.0	5.56–8.44	

ECOG scores^*∗*^
0–2	12	30.0	12	7.61–16.39	0.007
3–4	28	70.0	7	5.49–8.51	

Chemotherapy^*∗*^					
No	17	42.5	6.0	3.20–8.80	0.032
Yes	23	57.5	8.0	5.22–10.78	

Visceral metastasis^*∗*^					
No	8	20.0	12.0	9.849–14.15	0.002
Yes	32	80.0	7.0	5.87–8.13	

^*∗*^ *P*＜0.05, indicating statistical significance.

The article "Expression of CX3CL1 and CCL28 in Spinal Metastases of Lung Adenocarcinoma and Their Correlation with Clinical Features and Prognosis" was retracted in 2023. Reasons: suspected computer-generated content; unreliable results or conclusions; concerns about the data; concerns about the results or conclusions.

**Table 3:** Multivariate analysis of influencing patients' overall survival.

	B	Se	Wald	Df	Sig.	Exp (B)	95.0% CI exp (B)	
							Down	Up
Gender	−0.628	0.465	1.824	1	0.177	0.534	0.215	1.327
Age	−0.132	0.473	0.077	1	0.781	0.877	0.347	2.217
Number of bone metastases	0.570	0.629	0.823	1	0.364	1.769	0.516	6.065
ECOG scores	−1.085	0.692	2.455	1	0.117	0.338	0.087	1.313
Chemotherapy	0.805	0.502	2.569	1	0.109	2.236	0.836	5.982
Visceral metastasis	−0.983	0.737	1.777	1	0.182	0.374	0.088	1.587
CX3CL1^*∗*^	−1.264	0.627	4.067	1	0.044	0.283	0.083	0.965
CCL28	−1.621	0.901	3.235	1	0.072	0.198	0.034	1.156

^*∗*^ *P*＜0.05; OS, overall survival; HR, hazard ratio; 95% CI, 95% confidence interval.

## Data Availability

The datasets used and/or analyzed during the current study are available from the corresponding author on reasonable request.

## References

[1] Silbermann R. (2011). Introduction to the special issue on the microenvironment of bone metastasis. *Cancer Microenvironment*.

[2] Zhang Y., Zhao L., Wang X. (2018). Repopulating retinal microglia restore endogenous organization and function under CX3CL1–CX3CR1 regulation. *Science Advances*.

[3] Liang Y., Yi L., Liu P. (2018). CX3CL1 involves in breast cancer metastasizing to the spine via the Src/FAK signaling pathway. *Journal of Cancer*.

[4] Jarmin D. I., Rits M., Bota D. (2000). Cutting edge: identification of the orphan receptor g-protein-coupled receptor 2 as CCR10, a specific receptor for the chemokine ESkine. *The Journal of Immunology*.

[5] Shi S., Tao L., Song H., Chen L., Huang G. (2014). Synergistic antitumor effect of combining metronomic chemotherapy with adoptive cell immunotherapy in nude mice. *Acta Pathologica, Microbiologica et Immunologica Scandinavica*.

[6] Liu J.-F., Tsao Y.-T., Hou C.-H. (2017). Fractalkine/CX3CL1 induced intercellular adhesion molecule-1-dependent tumor metastasis through the CX3CR1/PI3K/Akt/NF-*κ*B pathway in human osteosarcoma. *Oncotarget*.

[7] Shulby S. A., Dolloff N. G., Stearns M. E., Meucci O., Fatatis A. (2004). CX3CR1-fractalkine expression regulates cellular mechanisms involved in adhesion, migration, and survival of human prostate cancer cells. *Cancer Research*.

The article "Expression of CX3CL1 and CCL28 in Spinal Metastases of Lung Adenocarcinoma and Their Correlation with Clinical Features and Prognosis" was retracted in 2023. Reasons: suspected computer-generated content; unreliable results or conclusions; concerns about the data; concerns about the results or conclusions.

[8] Gong L., Xu L., Yuan Z., Wang Z., Zhao L., Wang P. (2019). Clinical outcome for small cell lung cancer patients with bone metastases at the time of diagnosis. *Journal of Bone Oncology*.

[9] Sharma G. (2022). Chemokines network in bone metastasis: vital regulators of seeding and soiling. *Seminars in Cancer Biology*.

[10] Do H. T. T., Lee C. H., Cho J. (2020). Chemokines and their receptors: multifaceted roles in cancer progression and potential value as cancer prognostic markers. *Cancers*.

[11] Letourneur D., Danlos F.-X., Marabelle A. (2020). Chemokine biology on immune checkpoint-targeted therapies. *European Journal of Cancer*.

[12] Siegel R. L., Miller K. D., Jemal A. (2015). Cancer statistics, 2015. *CA: A Cancer Journal for Clinicians*.

[13] Aaron A. D. (1994). The management of cancer metastatic to bone. *JAMA: The Journal of the American Medical Association*.

[14] Jacobs W. B., Perrin R. G. (2001). Evaluation and treatment of spinal metastases: an overview. *Neurosurgical Focus*.

[15] De Bruyn P. P. (1981). Structural substrates of bone marrow function. *Seminars in Hematology*.

[16] Ribatti D., Mangialardi G., Vacca A. (2006). Stephen Paget and the ’seed and soil’ theory of metastatic dissemination. *Clinical and Experimental Medicine*.

[17] Ogihara S., Seichi A., Hozumi T. (2006). Prognostic factors for patients with spinal metastases from lung cancer. *Spine*.

[18] Wang Z., Ning L., Li H. (2014). Clinical observation of percutaneous osteoplas-ty in the treatment of 92 lung cancer patients with extraspinal bone me-tastases. *Tumor*.

